# Analysis of the Impact of the Development Level of Aerobics Movement on the Public Health of the Whole Population Based on Artificial Intelligence Technology

**DOI:** 10.1155/2022/6748684

**Published:** 2022-08-29

**Authors:** Weiping Ji, Xuan Qiu

**Affiliations:** ^1^College of Physical Education, Kunsan National University, Kunsan 54150, Republic of Korea; ^2^Department of Physical Education, Yichun University, Yichun 336000, China

## Abstract

With the enhancement of China's comprehensive national power and the improvement of people's living standards, health has become the goal that people pursue. While people are thirsty for extensive knowledge and a healthy body, they also pay more attention to the cultivation of elegant temperament and the enjoyment of beauty, and aerobics has become a hot spot for national fitness with its advantages of coordinated and beautiful movements, bright and cheerful rhythm and obvious fitness effects. Aerobics is a new popular fitness sports, from the beginning of development by most fitness enthusiasts, especially it is a women's favorite. To this end, the characteristics, value, status, and role of aerobics in the public health of all people are discussed, and the problems of poor recognition effect in the existing aerobics difficulty aerobics action recognition methods are proposed to apply the graph convolutional neural network to the aerobics difficulty aerobics action recognition. The video of aerobics is divided into several images, and the background of the aerobics difficult aerobics action image is eliminated, and the gray scale co-generation matrix is set to estimate the local area blur kernel of the difficult action image to correct the visual error of the difficult action image. “change to” The aerobics action is divided into several difficult action images, and the gray-scale symbiosis matrix is set to estimate the local area fuzzy core of the difficult action image, and correct the visual error of the difficult action image. On this basis, the graph convolutional neural network is pre-trained to construct a human-directed spatial-temporal skeleton map, and the human-directed spatial-temporal map representation is modeled with temporal dynamic information to achieve aerobics difficult aerobics action recognition. The experimental results show that the recognition time of the difficult aerobics movements based on the graph convolutional neural network is shorter and the number of false recognitions is less in complex and simple backgrounds, which proves that the proposed method improves the recognition of difficult aerobics movements to achieve the goal of promoting the development level of aerobics and improving the public health of all people.

## 1. Introduction

With the development of China's economy and the improvement of cultural living standards, the national demand for amateur cultural and sports activities has become more and more urgent, and fitness, leisure, and entertainment have gradually become the needs of people's daily life. Therefore, more and more people are actively involved in sports. At the same time, as China's national fitness program continues to promote and deepen, as well as by the influence of the Olympic Games, the enthusiasm of the masses to participate in sports activities has become unprecedentedly high [1–4]. As an emerging sport with a wide mass base, aerobics stands out among many traditional sports with its unique charm and is loved by more and more people. Its exercise intensity and movement difficulty are relatively low, and rich in content, diverse forms, easy to exercise, line effect is remarkable, can be used for different ages, levels, gender, occupation of the community. Whether in the public, scientific, or in the social, lifelong, diversity, etc., aerobics have incomparable superiority over other sports, and is the best way of public fitness. The development level of aerobics and the public health of the whole population are shown in Figure 1.

The role of aerobics in the national fitness movement, fitness role for the 21st-century Chinese sports advocate “people-oriented, health first” idea, pay attention to the health of the individual is the basis of public health, aerobics is in line with this multi-dimensional health values of the public sports and fitness projects [5–7]. Practice has proved that aerobic exercise can mostly develop the body's cardiorespiratory function, aerobics is a typical aerobic exercise, due to aerobics scientific and reasonable arrangements, so that all parts of the body through the exercise, to achieve a certain amount of load and practice density, the practitioner in a certain stage to maintain the intensity of exercise, and heart rate of 150 times/min, to get the effect of aerobic exercise. And it is rarely single joint local activities in each section of the exercise, mostly for multi-joint exercise, intensity from weak to strong, gradually increase the body load to maintain a certain amount of exercise and then gradually reduce so that the change in the heart rate of the exerciser from low to high, wave-shaped gradually rise, and then return to a calm state, so that the cardiovascular system, respiratory system, and other internal organs improve and strengthen the function and effective regulation of the body's internal environment.

Fitness comprehensive is the outstanding advantage of aerobics, and it is strictly in accordance with the anatomical parts of the human body, purposefully to achieve body proportion, coordination, bodybuilding development, and action design and choreography [8]. The whole set of movements is arranged from top to bottom, from left to right, both small joint movements, but also the day muscle group exercises, the body of the joints, various parts in the non-stop exchange of movement, so that people thoroughly do a whole-body exercise, to achieve the purpose of improving physical fitness. Most of these exercises are multi-joint synchronization, such as the waist, knee, ankle and head. Multi-joint synchronous movement not only increases the number of activities of the body joints but also can freely change the combination form and form a variety of movements, which is conducive to improving and enhancing the coordination of the body and achieving the effect of comprehensive exercise. A load of aerobics, mainly relies on the body parts of their own weight, through repeated exercises to achieve, so that the overall development of muscle strength, speed, and flexibility, improves the flexibility and flexibility of the joints, but also absorbed many hip movements in disco and jazz dance, both to improve the flexibility of the hip joint, but also to strengthen the often-neglected abdominal movement. The development of various qualities such as endurance and sensitivity also have a good impact on the human body's ability to adapt to the natural world and resistance to disease [9–11].

It can be said that aerobics is currently a more ideal exercise to improve the overall quality of the body. Practitioners can according to their different stages, different fitness purposes need to be targeted, sequential development of various parts of the body, so there are many fitness enthusiasts, aerobics as their lifelong sports activities. Cultivating people to develop the habit of lifelong physical activity is the goal pursued by national fitness. The realization of this goal will further promote the implementation of the national fitness program [12–15]. As the national fitness movement continues to deepen, people do not only pursue the recent fitness effect, but also pursue long-term multifaceted lifelong benefits. The content of aerobics is rich and inclusive. It does not stick to a certain dance material, where the healthy development of the body and the form of the dance can be compatible and order to blend into one.

It not only absorbs Chinese classical dance and martial arts movements but also boldly uses ballet movements, taking the beneficial components of the clever combination, in the beautiful music and rhythmic melody to do a large amplitude, strong sense of movement, and modeling of beautiful movements. Aerobics has a special effect on shaping the beauty of the body. Since the exercise intensity is small, exercise time is long, and the energy of long-time exercise mainly comes from the oxidation and decomposition of fat in the body, and often participate in the practice, it can effectively eliminate the body's excess fat, promote muscle firmness and plumpness, clear contour, soft and beautiful lines. The integration of national fitness and public health for all is the result of the development of the national economy and its compliance with the development of the trend of the times. The effective integration of national fitness and national public health can improve the physical and mental health of the public and meet the long-cherished wish of the public to increasingly pursue a better life. It is necessary to promote the effective integration of national fitness and national public health, and to integrate national public health into the development of all policies with the development goal of great health [16].

Sports aerobics action recognition is a research hotspot in the field of computer vision, which is widely used in visual surveillance, content analysis, paramedicine, intelligent human-computer interaction, and other fields. Among them, the field of aerobics also applies the recognition method of human body movements to improve the standard degree of aerobics movements, but the recognition is easily affected by the change of scene, the change of lighting, the difference of viewpoint and other factors, which leads to the poor recognition of aerobics movements in aerobics difficulties. For this problem, related researchers have conducted many studies [17–19]. The adaptive recognition method of aerobics decomposition action image based on feature extraction. The method uses the background small cut method for human target extraction, constructs binary image sequences of human contours, and uses the similarity detection method to decompose and match aerobics images to achieve the recognition of aerobics actions. Deep learning-based method for human aerobics action recognition in video. The method uses images and optical flow fields as inputs in the space and time domains and employs a decision fusion strategy for aerobics action recognition.

The main contributions of this study are as follows. For the analysis of the impact of the development level of aerobics on the public health of the whole population, the accuracy of aerobics action recognition can be improved by aerobics difficulty aerobics action recognition, and a method of aerobics difficulty aerobics action recognition based on graph convolutional neural network is proposed. The graph convolutional neural network is a feedforward neural network, artificial neurons in its coverage area of part of the surrounding units will produce a response, the texture, color and other features into the random forest and other classifiers, and then use the neural network to classify and complete the target feature extraction, based on this advantage of this network, it is applied to aerobics difficult aerobics action recognition, improve the recognition of aerobics difficult action, achieving an accurate analysis of the impact of the development level of aerobics on the public health of the whole population.

## 2. Related Work

### 2.1. The Current Situation of the Development of the Aerobics Movement

Aerobics is a kind of fitness exercise with high popularity in modern society. It is a combination of physical exercises and aerobic activities with a certain rhythm in a dance form accompanied by cheerful music. The sport of aerobics does not require a high degree of professionalism from the participants, so the public can quickly master the skills of aerobics through learning. Nowadays, people's requirements for physical health and quality of life are getting higher and higher, and the enthusiasm of the public to participate in social and cultural activities is also increasing. Aerobics has a certain role in improving body coordination, strengthening cardiorespiratory function, and exercising muscles, and the school is simple, so it is also loved by the people and widely carried out in social and cultural activities. The fitness value of aerobics exercise, aerobics exercise on the influence of physical beauty aerobics has an obvious bodybuilding function, through the training of aerobics, can help dancers form a good physical beauty, and can be effective in shaping and improving their body [20–22].

Compared with ordinary dance, aerobics has a stronger sense of rhythm and rhyme, and it incorporates a certain concept of movement, in the process of participating in aerobics, every joint of the body can get enough movement, which is in line with the current requirements of sports and fitness. When participants adhere to a period of aerobics exercise, limbs will be more flexible, the body's reaction speed will also become faster, through the aerobics exercise can make the body fat burning, help slim body. Long-term participants in aerobics exercise, their waist, and back more strength, and almost no fat and belly, not only the shape becomes more beautiful, but also the body will become healthier [23]. Nowadays, the pace of life is accelerating, young people work under pressure and have little time to participate in fitness training, making many young people generally have lower physical fitness. By regularly participating in aerobics, the flexibility of dance movements and the balance of sports can be used to promote the improvement of the dancer's body coordination ability. Aerobics has a variety of forms of movement, which can make dancers' waist, back, shoulder, knee joints, cervical spine, etc, whole-body joints exercise at the same time. Aerobic exercise can effectively improve the body flexibility of dancers.

At present, Chinese residents generally decline in physical quality, the incidence of arthritis and rheumatic bone pain diseases is very high, and not limited to the elderly, many young people have different degrees of cervical spondylosis, rheumatism, etc. Therefore, to actively promoting the concept of national fitness, more people should participate in aerobics, as it increase the flexibility of the limbs and improve the quality of life, so that we can feel a more beautiful life [24]. Under the heavy work pressure and life stress, insomnia, dreaminess, neurasthenia, and other diseases seem to have become the typical diseases of modern people, and the incidence of Alzheimer's, stroke and other brain function diseases are increasing year by year. Aerobics requires learning different dance movements, and to follow the rhythm of the music for body movements, in order to ensure coordination with the rhythm and the standard of body movements, it is necessary to remember and coordinate through their own brain, this process can be through frequent brain activity, exercise the brain function of dancers, so that their brain to maintain vitality, and to maintain a fast reaction speed, in this case, it will be less prone to memory loss, neurasthenia and other degenerative phenomena.

To exercise the brain function more effectively, improve the coordination ability between brain and body. You can use cardio as a daily exercise to get a healthy body. The whole-body exercise promotes blood circulation, and improve the oxygen supply capacity of the blood, as well as tbrings a a good impact on the brain to a certain extent. The flexibility of the brain thinking and memory, learning ability, and other aspects of people who exercise regularly will certainly be much better than those who do not exercise regularly.

### 2.2. Public Health for All People

Health is an inevitable requirement for the promotion of all-around human development, a basic condition for economic and social development, an important symbol of national prosperity and national wealth, and a common pursuit of the public. To achieve the strategic goal of a healthy China, prevention should be the focus, indicating the important position of preventive health care in the improvement of the public health of the whole population, and also putting forward higher requirements for the improvement of national health literacy [25].

Health literacy, as an important component of human capital, contains both cognitive and non-cognitive abilities related to health. The improvement of health literacy not only significantly improves the health status of individuals, but also enhances the health benefits of the surrounding people and the whole society, with positive spillover effects. Therefore, in the long term, health literacy is an important determinant of improving the health behaviors of a country's population and enhancing overall health. In the context of the global pandemic of New Coronary Pneumonia, health literacy as a long-neglected determinant of health has attracted widespread attention worldwide. Studies have found that residents with higher health literacy are able to understand virus knowledge and epidemic prevention information more accurately, establish correct knowledge of the epidemic, and take effective epidemic prevention measures. Therefore, as China implements a normalized epidemic prevention and control policy, improving national health literacy is important to continuously consolidate the prevention and control achievements of the new crown pneumonia epidemic [26]. Meanwhile, as China's population ages and people's lifestyles change, the burden of chronic non-communicable diseases such as cardiovascular diseases and cancer continues to increase, and health literacy plays a crucial role in disease prevention and control, chronic disease management, and effective use of medical resources. Based on the above research findings, the author makes the following policy recommendations to improve the health literacy of Chinese residents and serve the health China strategy.

Emphasize health education in schools and further strengthen health science in primary and secondary school campuses. Education is important for improving health literacy, and the questionnaire results show that individual education level has a significant positive effect on health literacy scores, and this effect is reflected in all dimensions of health literacy. This is because education plays an important role in the formation and early accumulation of health literacy. On the one hand, education can enhance individuals' cognitive abilities in word reading, mathematical calculation, and other aspects, thus providing a cognitive foundation for the acquisition, recognition, understanding, and application of health knowledge; on the other hand, education has an important role in shaping minors' behavioral habits, interpersonal communication, and other non-cognitive abilities, thus bringing about a healthy lifestyle and medical habits when individuals become adults important impact. By organically integrating health science with knowledge learning in schools at an early stage of students' growth, we can help minors establish correct health concepts and develop good health habits early on, thus having a better foundation for health literacy. Paying attention to the importance of preventive health care in the improvement of the public health level of the whole population, it is especially necessary to pay attention to and strengthen the scientific popularization of disease prevention among middle-aged groups [27].

Currently, sub-health problems and a high risk of chronic diseases are prevalent among workers in major Chinese cities. The high-intensity work pace, unhealthy lifestyle, and the high prevalence and youthfulness of chronic diseases have put considerable pressure on the health benefit improvement of the whole society. In addition, insufficient awareness of infectious disease prevention can lead to difficulties for individuals to respond effectively to sudden public health events such as the New Coronary Pneumonia outbreak, leading to increased load on medical institutions and crowding out of medical resources, to the detriment of overall prevention and control. With the overall development of China's economy and the continuous promotion of the commonwealth, the central and western regions are bound to pay more attention to disease prevention and health care in the future, and the demand for and attention to health literacy will gradually grow. Therefore, increasing health promotion and popularization in the central and western regions (especially the less developed regions) is of great significance to narrow the gap in health literacy levels between regions and achieve the common improvement of public health.

### 2.3. Artificial Intelligence Technology

Nowadays, aerobics action recognition technology is widely used in various fields, such as surveillance, games, and human-computer interaction. Among different aerobics action recognition methods, human skeleton-based aerobics action recognition has the characteristics of small data set size, unaffected by lighting, good structural information compared with RGB video-based human aerobics action recognition, and the former can be combined with the latter mutually [28–30]. Therefore, human skeleton-based aerobics action recognition has also gradually become a hot spot for current research. Among them, human skeletal data is a skeletal sequence consisting of 2D/3D coordinates of joints in several frames and is temporal in nature. In the task of aerobics movement recognition, how to extract more distinguishing features is the focus and the difficulty.

In the field of human skeletal aerobics movement recognition, deep learning methods have certain superiority over manual feature methods. Therefore, human skeletal aerobics movement recognition based on deep learning methods, such as convolutional neural network, recurrent neural network, and graph convolutional neural network, has been widely used in human skeletal aerobics movement recognition tasks. The early network frameworks for human skeletal aerobics movement recognition are mainly CNN and RNN. a hierarchical co-occurrence network based on CNN to achieve the extraction of global joint co-occurrence features and achieved good results at that time; the importance of joint spatial configuration, a dual-stream recurrent neural network based on RNN is proposed to extract joint spatial features and time-dependent features respectively. Although both CNN and RNN can be used for aerobics movement recognition tasks based on human skeleton, the important information of the graphical structure of the human skeleton is neglected. With the rise of GCN, GCN has started to be combined with human skeletal aerobics movement recognition.

GCN is applied to the human skeletal aerobics movement recognition task, using the physical structure features of human skeleton for spatial-temporal modeling, proposing a spatial-temporal graphical convolutional neural network and providing ideas for the next research. Action structure graph convolutional neural networks are proposed for how to capture potential joint correlations, and the skeleton graph is extended on top of that so that higher-order joint dependencies can be represented. The fixed graph topology of the human skeleton affects the training and performance of the model, so a dual-stream adaptive graph convolutional neural network is proposed, which uses a combination of fixed and non-fixed graph topologies to increase the graph flexibility and introduce second-order skeletal information.

The multi-scale aggregation of cross-temporal graphs is used to learn joint features and skeletal features separately in a dual-stream network with a multi-scale unified spatial-temporal graph convolutional network with dual streams. Considering the importance of potential information in the 3D skeleton and how to encode it, a spatial-temporal converter network is proposed to capture the correlation of different factions within frames by a spatial converter and inter-frame correlation using a temporal converter, and a dual-stream network model is constructed to combine both converters. The non-physical correlations between joints are captured by regionally correlated graph convolution and the second-order skeletal information is used to propose a regionally correlated adaptive graph convolution neural network. Although all the above methods achieve good results, they generally pay attention to the recognition accuracy of the model and ignore the efficiency problem of the model. Therefore, the semantic-guided neural network with one-hot encoding introduces high-level semantics to reduce the number of parameters and computation of the model. The Ghost module is introduced to reduce the number of parameters and computation of the model, and the single-stream network is used to further reduce the number of parameters of the model, and multiple information is introduced into the model by direct merging fusion, and the non-local Ghost graph convolutional network is proposed.

## 3. Methods

### 3.1. Model Architecture

The assisted virtual training motion detection system designed in this study consists of three layers: the logic layer, the technology layer, and the application layer. The overall structure of the system is shown in Figure 2. As can be seen from Figure 2, the logic layer of the system is mainly responsible for collecting training behavior data and processing them accordingly to obtain action detection results; the technology layer mainly includes relevant technologies applied for processing training action techniques; the application layer is mainly responsible for storing the initial image data and processed image data, and the interactive interface displays the virtual training actions. This system uses intelligent services as the carrier of framework construction, which can effectively improve the detection performance of the system.

### 3.2. Aerobics Action Pre-Processing

To realize the recognition of aerobics difficult movements, the video image of aerobics movements needs to be analyzed first. The video contains many aerobics movements, the length of the movements varies, and the same movements can have differences. Therefore, the aerobics video needs to be divided into several images. The divided action images are pre-processed using the energy pyramid method. In this process, the multilayer pyramid structure of action images is constructed, the temporal pyramid energy histogram is obtained, and then the pyramid of each layer is solved, and the calculation formula is expressed as:

(1) $$\begin{array}{c} Q\left(i\right)=\frac{\sum_{i}^{j=1}\sum r\left|L_{r}^{i}/L_{r}^{i}+\delta \right|}{\sum_{n}^{j=1}\sum r\left|L_{r}^{i}/L_{r}^{i}+\delta \right|}. \end{array}$$

In formula, *r* represents the amplitude threshold of the aerobics motion image, *L*_*r*_^*i*^ represents the aerobics difficulty action depth image sequence, and *δ* represents the aerobics action angle value. The above processing method can store the aerobics image sequence into each level of the pyramid, based on which the inter-frame differencing method is used to eliminate the background of the image. The specific algorithm of the inter-frame difference method is to subtract the two frames after grayscale transformation to obtain the difference between each pixel point, which is calculated as follows:

(2) $$\begin{array}{c} D\left(x,y\right)=\left\{\begin{array}{cc} 1, & \text{if}\left|f_{k-1}\left(x,y\right)-f_{k}\left(x,y\right)\right|>T,\\ 0, & \text{others.} \end{array}\right. \end{array}$$

In the formula, 1 corresponds to all the pixel points that changed during the calculation, 0 represents the pixel points that did not change during the detection process, *f*_*k*−1_(*x*, *y*), *f*_*k*_(*x*, *y*) both represent the detection image, and *T* represents the threshold value. Through the above process, the aerobics video is divided into images and the background elimination process is done on the images, which provides the basis for aerobics difficulty aerobics movement recognition.

### 3.3. Image Visual Error Correction

Based on the pre-processing of the above aerobics action video images, the visual error correction of the aerobics difficult action images is done as follows. The grayscale co-generation matrix is set to analyze the aerobics action image texture, and the spatial distribution state of image pixels is described to obtain.

(3) $$\begin{array}{c} f\left(x,y\right)=f_{ij}\left(x+a,y+b\right). \end{array}$$

In equation, *f*_*ij*_ is the *i*, *j* pixel proximity state, *a* represents the length in the *x* direction, and *b* represents the length in the *y* direction, respectively. Estimating the local region fuzzy kernel of the aerobics image, after the above processing, the action image pixel intensity and gradient are used as the a priori knowledge of the fuzzy kernel to solve the degree of recovery of the whole action image, and the calculation formula is expressed as:

(4) $$\begin{array}{c} P\left(x\right)=\sigma P_{t}\left(x\right)+P_{t}\left(\nabla x\right). \end{array}$$

In equation, *P*_*t*_(*x*) represents the number of non-zero-valued pixels, *P*_*t*_(∇*x*) represents the gradient value of pixels, *P*(*x*) represents the prior knowledge, and *σ* is the weighting factor. Motion image visual error correction. There is a certain error between the visual image and the original aerobics image, which needs to be further processed, i.e.

(5) $$\begin{array}{c} I=\hat{I}+E. \end{array}$$

In equation, $\hat{I}$ represents the visual image and *E* is the error image. On this basis, the optimal estimation is performed, and the expression is expressed as

(6) $$\begin{array}{c} {\hat{E}}_{K}=g_{b}\left(E\right). \end{array}$$

In equation, *g*_*b*_ is the difference operator and *E* represents the image error. The error correction of the aerobics action image by the above process provides the basis for the identification of aerobics difficult aerobics actions.

### 3.4. Convolutional Neural Network

The graph convolution structure is shown in Figure 3. The convolution layer, as the core part of the network, mainly performs the convolution calculation of the aerobics difficulty action feature map to obtain more abstract image features. The method obtains different output feature maps by performing convolutional calculations on the input data of the previous layer within this layer, which is expressed by the formula:

(7) $$\begin{array}{c} y_{mn}=f\left(\sum^{Q-1}\sum^{P-1}x_{m+i,n+j}w_{ij}+b\right). \end{array}$$

In equation, *x*_*m*+*i*,*n*+*j*_ represents the image pixel value of point, *w*_*ij*_ represents the weight value of the convolution kernel size on point (*i*,*j*), *b* represents the bias size of this layer, *f* represents the network activation function, and *Q* and *P* represent the image resolution size parameters, respectively. Pooling layer: This layer mainly reduces the resolution of the feature map and accelerates the speed of aerobics difficulty aerobics action recognition, and the pooling operation process is as follows.

(8) $$\begin{array}{c} y_{mm}=f\left(w\frac{1}{S_{1}S_{2}}\sum_{S_{2}-1}^{j=0}x_{m\times s_{1}+i,n\times S_{2}+j}+b\right). \end{array}$$

In equation, *x*_*m*×*s*_1_+*i*,*n*×*S*_2_+*j*_ represents the pixel value of the input data at the point, and *y*_*mm*_ represents the output value after the pooling operation. To achieve the best fit for parameters such as weights and biases in the network, it is also necessary to construct a multi-level computational model with the following formula.

(9) $$\begin{array}{c} h_{w,b}\left(X\right)=f\left(\sum_{n}^{i=1}w_{i}x_{i}+b\right). \end{array}$$

In equation, *X* is the input vector, *w*_*i*_ and *x*_*i*_ represent the bias parameters of the *i*th data, respectively, and *b* represents the activation function. Then, multiple consecutive frames are superimposed in the convolution layer, and multiple consecutive frames are sequentially passed through the convolution layer to generate multiple sequences of adjacent consecutive frame strings in the previous layer.

(10) $$\begin{array}{c} v_{ij}^{xyz}=\left(b_{ij}+\underset{m}{\sum }\overset{p=0}{\underset{K}{\sum }}\overset{r=0}{\underset{p}{\sum }}\right). \end{array}$$

In equation, *b*_*ij*_ represents the deviation of the *j*-th feature map in the *i*th layer, *m* represents the number of feature maps, *K* represents the spatial dimensional size parameter, and *p* represents the convolutional kernel weights. The above process pre-trains the network so that the neural units in the network are connected, which in turn can be directly input to the image and facilitate the processing of image data.

### 3.5. Directed Spatial-Temporal Skeleton Map of Human Body

The original skeleton data are column frames, each frame contains a set of human joint coordinates, to accurately identify the difficult movements of aerobics, the human body is constructed as a directed spatial-temporal skeleton map. The skeletal information is extracted according to the 2D or 3D coordinates of the joints to construct an adaptive directed acyclic map. Taking the 3D skeleton data as an example, the joints sitting in the original data are labeled as (*x*, *y*, *x*), and given a skeleton, and the target joint is represented as *v*, the vector of the skeleton is represented as:

(11) $$\begin{array}{c} E_{v_{s},v_{s}^{\prime }}=\left(x_{s}-x_{s}^{\prime },y_{s}-y_{s}^{\prime },z_{s}-z_{s}^{\prime }\right). \end{array}$$

Traditional methods of modeling skeletal data ignore the kinematic dependence between joints and bones, and in this study, the human skeleton is represented as a directed acyclic graph. The points of the joints are used as vertices, the bones are used as edges, and the direction of each skeletal edge is determined by the relationship between the joint point and the root node. The above process represents the skeleton structure as a directed graph, which provides the basis for extracting the information in the graph.

### 3.6. Human Directed Spatial-Temporal Graph Representation

A directed graph is constructed using a directed graph neural network, which consists of multiple graph layers populated with graphs with vertex and bone attributes between each layer, capable of propagating information in adjacent joints and bones, and capable of updating their association information between layers and outputting graphs with updated attributes. In each layer, attributes are updated based on adjacent edges and vertices, and in each layer, vertices and edges receive attribute information from adjacent edges or vertices. Two aggregation functions are mainly used for the expression of multiple incoming and outgoing edge attributes of the vertex, due to the existence of more centripetal and centrifugal points in the root node, that is, there are multiple input and output edges as well as multiple sources and target nodes, for this reason, the propagation formula of information is established according to the input and output edges of the root node, the calculation formula is expressed as:

(12) $$\begin{array}{c} e_{i}^{\text{in}}=\sum_{k}^{k=1}\left(\frac{\alpha_{k}}{\sum_{k}^{k=1}\alpha_{k}}\right)g^{\text{in}}\left(R_{ik}^{\text{in}}\right),\\ e_{i}^{\text{out }}=\sum_{k}^{k=1}\left(\frac{\alpha_{k}}{\sum_{k}^{k=1}\alpha_{k}}\right)g^{\text{out}}\left(R_{ik}^{\text{out}}\right). \end{array}$$

In equation, *α*_*k*_ represents the correlation of samples between the root node and centripetal and centrifugal points, i.e., the human skeleton action co-relation parameter; *g*^out^ represents the aggregation function of the output edge, *R*_*ik*_^out^ represents the aggregated output result, and *R*_*ik*_^in^ represents the aggregated input function. To learn the co-occurrence relationship between human skeleton adaptively, *α*_*k*_ is represented by two fully connected layers of learning, the first one is activated by a nonlinear function, and the second one is a SoftMax layer, which is used to learn the correlation between root nodes and centripetal points. If both co-occurring root nodes and non-cooccurring correlation nodes are present in an action, the correlation nodes between these two actions are calculated.

(13) $$\begin{array}{c} A_{v}=\left[\begin{array}{ccc} 1 & 1 & 0\\ 0 & 1 & 0\\ 1 & 1 & 1 \end{array}\right],\\ A_{r}=\left[\begin{array}{ccc} \alpha_{i1} & 0 & 0\\ 0 & 1 & 0\\ \alpha_{i4} & \alpha_{i5} & 0 \end{array}\right]. \end{array}$$

There are three rows in the nodal-directed matrix *A*. The first row is the group of centripetal nodes, where 0 represents no connection and 1 represents the source node; the second row is the root node and the third row represents the group of centrifugal nodes, where 1 represents the target node and 0 represents no connection.

## 4. Experiments and Results

### 4.1. Experiment Setup

The experimental data was obtained from non-public data of an aerobics research institute in China, and was conducted in two scenes, the first part of the experiment was shot in a fixed background with aerobics movements; the second part was shot in an actual scene, which contained lighting information, partial occlusion, camera movement, and other situations. A total of 100 images are selected from the captured videos, respectively, and a total of ten experiments are conducted, with 10 images recognized in each experiment and their averages were taken. The recognition effects of the proposed method, recognition method based on feature extraction and recognition method based on deep learning are compared in the two scenarios. Experimental platform. The graphics card is a single NVIDIA RTX 2060 Super, the processor is Intel i5 9400F, the memory is 32 GB, the operating system is Ubuntu 19.04, the language is Python 3.7, the CUDA version is 10.2, and the PyTorch 1.4.0 framework is used. The relevant parameters are set. To make the feature map size of each layer convolution match the multi-channel adaptive map size, the number of frames of the skeletal sequence is set to 25 in this paper, and the number of channels in the network C1 to C4 are 64, 128, 256, and 512, respectively. In this paper, in order to compare the baseline method more fairly, other hyperparameters are set the same as the baseline method, and the Adam optimizer is used, with the initial learning rate of 0001, a weight decay value of 0.0001, a number of loaded data threads of 16, a training period of 120 epochs that decreases by a factor of 10 at 60, 90, and 110 cycles, respectively, and a batch size of 64 for training and 32 for testing. dataset settings. The dataset was set up using two recommended evaluation settings, namely CS (cross-topic) and SS (cross-setting number). To make the model more generalizable, the same data setup method as the baseline method is adopted in this paper, where the 3D skeletons in each sequence are randomly rotated by a certain angle around the *X*, *Y* and *Z* axes, respectively. For the data pre-processing part, the random pool data pre-processing method proposed in this paper is used. Training time. The model was trained on a single NVIDIA RTX 2060 Super graphics card using the NTU RGB + *D* 120 dataset, and the total time taken to train the full 120epoch in each evaluation setup was more than 2 hours. The training process performance enhancement and loss convergence are shown in Figures 4 and 5.

### 4.2. Experimental Results

The results of the comparison of the aerobics movement recognition effect in simple backgrounds, the results of the comparison of the aerobics movement recognition time of the three methods in simple backgrounds are shown in Figure 6. By analyzing Figure 6, we can find that the studied method spends less time on aerobics movement recognition than the other two methods.

The number of aerobics movement recognition errors for the three methods in a simple context is compared, as shown in Table 1. Analyzing the data in Table 1, it can be found that the studied method of aerobics difficult aerobics movement recognition based on graphical convolutional neural network does not have any false recognition in the simple background. Both the feature extraction-based recognition method and the deep learning-based recognition method have different numbers of false recognition cases. In contrast the recognition effect of the studied recognition method is better.

The results of the comparison between the proposed aerobics difficulty aerobics recognition method and the other two methods in the complex background are shown in Figure 7. Analysis of Figure 7 shows that the proposed aerobics difficulty aerobics recognition method takes the least time, while the other two methods take more recognition time, which is significantly more than the simple background aerobics movement recognition time. The recognition time is significantly more than that of the simple background aerobics movements, and the recognition efficiency is poor.

Analyzing the data in Table 2, the number of recognition errors of the three aerobics movement recognition methods in the complex background is significantly more than that in the simple background, but the studied aerobics movement recognition methods have fewer cases of false recognition. The recognition methods based on feature extraction and recognition methods based on deep learning increase the number of recognition errors more, and the recognition effect is worse.

In summary, the studied aerobics difficulty aerobics movement recognition method has less error recognition in simple and complex backgrounds and takes less time, which is better than the application of the other two methods. The reason is that the aerobics difficult aerobics action recognition method in this study preprocesses aerobics images and uses graph convolutional neural network to do multi-step recognition of actions, thus improving the recognition of aerobics difficult actions.

To verify the effectiveness of the random pool data pre-processing method proposed in this study, both the method and SGN model are experimented with using different data pre-processing methods. For a fair comparison, the skeletal sequence length was set to 25 in both data pre-processing methods. ODP indicates the use of the data pre-processing method, and NDP indicates the use of the random pool data pre-processing method in this paper. The experimental results in Figures 8 and 9 show that the recognition accuracy is improved by 4.2% on the CS evaluation settings and 3.1% on the SS evaluation settings when the SGN model is used, and by 3.7% on the CS evaluation settings and 3.4% on the SS evaluation settings when the LMI-GCN model of this paper is used. The reason for the improvement of model recognition accuracy is that the random pool data pre-processing method in this paper can effectively solve the problem of losing some skeletal sequence frames caused by data pre-processing, avoiding the loss of some important information, and further increasing the randomness of the data set, so that the model can learn more important distinguishing features and increase the model generalization.

In Table 3, (-G) indicates that no multi-channel adaptive map is used. The experimental results in Table 3 show that eliminating the multi-channel adaptive map causes the graph convolution in the model to degenerate into ordinary convolution, which is unable to aggregate the nodal features with relevance, thus leading to the degradation of the model performance. Compared with the model with the elimination of multi-channel adaptive map, the recognition accuracy of the model with multi-channel adaptive map is improved by 2.4% on CS evaluation settings and 2.6% on SS evaluation settings.

## 5. Conclusion

In summary, aerobics has distinctive features and comprehensive effectiveness, and has many favorable conditions for the promotion. Aerobics has low requirements for venue equipment, which is suitable for the current situation of China's stadium facilities and for the current situation of China's national and personal sports investment, in line with the national conditions; it is easy to disseminate and instruct, simple to learn and easy to promote; it is suitable for different groups, with a wide promotion area and easy to popularize; it has a high exercise value, which can comprehensively enhance people's physical fitness, regulate their psychology and improve their mental outlook, in line with the public's coordinated physical and mental development It meets the needs of the public's pursuit of beauty and is liked by the public. Aerobics in China already has a certain mass base, if you strengthen the propaganda, correct guidance, accelerate the training of aerobics instructors, pay attention to the creation of aerobics, through television and other means of comprehensive promotion. Aerobics can definitely play a special role in China's national fitness movement.

Aerobics is an important way and means to achieve the public health of all people through reasonable and scientific sports to promote the public health of all people. Residents' universal public health literacy is influenced by multiple factors such as age, gender, work, income, and education, showing different levels, respectively, and there are significant differences in the mastery of three aspects: basic knowledge and concepts of universal public health literacy, universal public health lifestyles and behaviors, and universal public health skills. In this study, we proposed an AI-based analysis model of the influence of the development level of aerobics on universal public health to determine the path of universal public health literacy improvement and effectively guarantee the physical and mental universal public health of residents. In the future, we plan to carry out research on the analysis of the impact of the development level of aerobics on the public health of the whole population using recurrent neural networks.

## Figures and Tables

**Figure 1:** The development level of aerobics and the public health of the whole population.

**Figure 2:** Model structure.

**Figure 3:** Graph convolution structure.

**Figure 4:** Schematic diagram of training process performance improvement.

**Figure 5:** The training process loss convergence schematic.

**Figure 6:** Action recognition time comparison in simple background.

**Figure 7:** Action recognition time comparison under complex background.

**Figure 8:** CS comparison of random pool data pre-processing methods.

**Figure 9:** SS comparison of random pool data pre-processing methods.

**Table 1:** Comparison of the number of action recognition errors in a simple context.

Number of experiments/times	Number of times the recognition method studied in a simple context was incorrectly recognized (time)	Number of false recognitions of recognition methods based on feature extraction in a simple context (time)	Number of false recognitions of recognition methods based on deep learning in a simple context
1	0	2	3
2	0	2	2
3	0	2	2
4	0	1	2
5	0	3	2
6	0	2	4
7	0	3	2
8	0	3	0
9	0	4	0
10	0	2	1

**Table 2:** Comparison of the number of action recognition errors in complex backgrounds.

Number of experiments (times)	Number of times the recognition method studied in a simple context was incorrectly recognized (time)	Number of false recognitions of recognition methods based on feature extraction in a simple context (time)	Number of false recognitions of recognition methods based on deep learning in a simple context
1	1	5	8
2	0	6	8
3	0	5	9
4	0	6	6
5	1	6	8
6	0	8	7
7	0	9	7
8	0	9	8
9	0	6	8
10	0	4	7

**Table 3:** Comparison of the effectiveness of multi-channel adaptive maps.

Algorithm	Param (*M*)	CS (%)	SS (%)
LMI-GCN (-G)	0.57	83.6	82.2
LMI-GCN	0.61	84.6	86.2

## Data Availability

The datasets used during the current study are available from the author on reasonable request.

## References

[1] Zhao M., Chen C., Liu L., Lan D., Wan S. (2022). Orbital collaborative learning in 6G space-air-ground integrated networks. *Neurocomputing*.

[2] Chen C., Zeng Y., Li H., Yangyang L., Shaohua W. (2022). A multi-hop task offloading decision model in mec-enabled internet of vehicles. *IEEE Internet of Things Journal*.

[3] Chen C., Li H., Li H., Fu R., Liu Y., Wan S. (2022). Efficiency and fairness oriented dynamic task offloading in internet of vehicles. *IEEE Transactions on Green Communications and Networking*.

[4] Chen C., Jiang J., Zhou Y., Lv N., Liang X., Wan S. (2022). An edge intelligence empowered flooding process prediction using Internet of things in smart city. *Journal of Parallel and Distributed Computing*.

[5] Chen C., Jiang J., Fu R., Chen L., Cong L., Shaohua W. (2021). An intelligent caching strategy considering time-space characteristics in vehicular named data networks. *IEEE Transactions on Intelligent Transportation Systems*.

[6] Lai Y., Zhang L., Han D., Zhou R., Wang G. (2019). Fine-grained emotion classification of chinese microblogs based on graph convolution networks. *World Wide Web*.

[7] Guo K., Hu Y., Qian Z. (2020). Optimized graph convolution recurrent neural network for traffic prediction. *IEEE Transactions on Intelligent Transportation Systems*.

[8] Li J., Liu L., Minami I., Miyagawa S., Sawa Y. (2021). Fabrication of thick and anisotropic cardiac tissue on nanofibrous substrate for repairing infarcted myocardium. *Methods in Molecular Biology*.

[9] Zhou H., Zhang F., Du Z., Liu R. (2021). Forecasting PM2.5 using hybrid graph convolution-based model considering dynamic wind-field to offer the benefit of spatial interpretability. *Environmental Pollution*.

[10] Qin L., Che W., Ni M. (2021). Knowing where to leverage: context-aware graph convolution network with an adaptive fusion layer for contextual spoken language understanding. *IEEE/ACM Transactions on Audio, Speech, and Language Processing*.

[11] Zhai R., Zou J., He Y. (2022). IAGC: interactive attention graph convolution network for semantic segmentation of point clouds in building indoor environment. *ISPRS International Journal of Geo-Information*.

[12] Li G., Knoop V. L., van Lint H. (2021). Multistep traffic forecasting by dynamic graph convolution: interpretations of real-time spatial correlations. *Transportation Research Part C: Emerging Technologies*.

[13] Wu S., Fei H., Ren Y., Li B., Li F., Ji D. (2021). High-order pair-wise aspect and opinion terms extraction with edge-enhanced syntactic graph convolution. *IEEE/ACM Transactions on Audio, Speech, and Language Processing*.

[14] Zhou G., Chen W., Li X., Qianshan G., Lizhe W. (2021). Split depth-wise separable graph-convolution network for road extraction in complex environments from high-resolution remote-sensing images. *IEEE Transactions on Geoscience and Remote Sensing*.

[15] Kearnes S., Mccloskey K., Berndl M., Pande V., Riley P. (2016). Molecular graph convolutions: moving beyond fingerprints. *Journal of Computer-Aided Molecular Design*.

[16] Batrak A. S., Polyakova A. V. (2013). Water aerobics as a form of health activities. *European Journal of Physical Education and Sport*.

[17] Pashkovskaya Y. (2013). Technique of carrying out the health-improving aerobics training session taking into account the somatotype of girls aged 11–13 years. *Uchenye Zapiski Universiteta Imeni P F Lesgafta*.

[18] Ross L. M., Barber J. L., Sui X., Blair S. N., Sarzynski M. A (2017). Abstract 37: the association of cardiorespiratory fitness and ideal cardiovascular health in the aerobics center longitudinal study. *Circulation*.

[19] Feng D., Huang K., Lan T. (2017). Influence model of health effect of aerobics exercise for college students. *Revista de la Facultad de Ingenieria*.

[20] Lemetti H., Jasinski T., Taim L., Tammaru M. (2013). PARE0001Tartu rheumatism association: “Physical activity and water are beneficial for joint health”. Hele lemetti, tiina jasinski, lea taim, marika tammaru. *Annals of the Rheumatic Diseases*.

[21] Jacqui W. (2016). Swimming, aerobics, and racquet sports are linked to lowest risk of cardiovascular death. *BMJ*.

[22] Bahram M. E., Akkasheh G., Akkasheh N. (2014). Aerobics, quality of life, and physiological indicators of inactive male students’ cardiovascular endurances, in Kashan. *Nursing and Midwifery Studies*.

[23] Dunsky A., Yahalom T., Arnon M., Lidor R. (2017). The use of step aerobics and the stability ball to improve balance and quality of life in community-dwelling older adults-a randomized exploratory study. *Archives of Gerontology and Geriatrics*.

[24] Jasiński R., Socha M., Sitko L., Kubicka K., Wozniewski M., Sobiech K. A. (2015). Effect of nordic walking and water aerobics training on body composition and the blood flow in lower extremities in elderly women. *Journal of Human Kinetics*.

[25] Li L. S. (2013). Establishment and analysis of the SPSS based regression model on aerobics regarding mid-aged and young women. *Applied Mechanics and Materials*.

[26] Lee T. E. (2013). Effects of aerobics intervention on health-related physical fitness and exercise behavior of the middle-aged and elderly people. *International Journal of Sport and Exercise Science*.

[27] Bryukhanova N. A., Bulgakova O. V., Mokrova T. I., Bogashchenko Y. A. (2013). Determination of possibilities of the use of high-intensive trainings facilities on lessons health aerobics. *Physical Education of Students*.

[28] Pivneva M. M., Rumba O. G. (2013). Aerobics health as means of increasing somatic health of students of special medical group. *Pedagogics Psychology Medical Biological Problems of Physical Training & Sports*.

[29] Liu Z., Liu Z., Fu X. (2021). Dynamic origin-destination flow prediction using spatial-temporal graph convolution network with mobile phone data. *IEEE Intelligent Transportation Systems Magazine*.

[30] Shen G., Zhao Z., Kong X. (2021). GCN2CDD: a commercial district discovery framework via embedding space clustering on graph convolution networks. *IEEE Transactions on Industrial Informatics*.

